# Personalized Item Recommendation Algorithm for Outdoor Sports

**DOI:** 10.1155/2022/8282257

**Published:** 2022-07-31

**Authors:** Hao Lei, Xinru Shan, Liwei Jiang

**Affiliations:** ^1^Department of Physical Education, Zhongnan University of Economics and Law, Wuhan 430073, Hubei, China; ^2^Department of Physical Education, Huazhong Agricultural University, Wuhan 430070, Hubei, China; ^3^Administration Office, China University of Geosciences Wuhan Future City Campus, Wuhan 430074, Hubei, China

## Abstract

With the rapid development of China's economy, people are eager for an effective way to relieve work pressure and strengthen their health at the same time. Outdoor sport is one of the best choices for people. However, the amount of recommended data on the network is very large. As a result, when people understand outdoor sports through the network, they cannot effectively obtain the information they want. This is the problem of “information overload,” and personalized recommendation system can effectively alleviate this problem. In order to effectively recommend outdoor sports to users, a useful attempt was made in the personalized recommendation system for outdoor sports in this paper. The specific work of this paper is as follows: firstly, the current situation of outdoor sports in China was summarized, and the related technologies of the recommendation system were studied, including user modeling technology, recommendation target modeling technology, and recommendation algorithm. In order to obtain better recommendation effect, this paper proposes to mix user-based collaborative filtering recommendation algorithm, project-based collaborative filtering recommendation algorithm, and content-based recommendation algorithm. The hybrid algorithm adopts the way of feature expansion and weighted combination. Firstly, the hybrid model (model 1) of user-based collaborative filtering recommendation and content-based recommendation is obtained. Secondly, the hybrid model (model 2) based on project collaborative filtering recommendation and content-based recommendation was obtained. Finally, model 1 and model 2 were combined together to get a hybrid model with better final recommendation effect. For the common cold start problem in the recommendation system, the system adopts content-based recommendation algorithm to solve it.

## 1. Introduction

With the rapid development of China's economy, the competition in various industries is becoming more and more fierce, the pace of society is becoming faster and faster, the work pressure is increasing, and the overtime situation in some industries is more serious. People live in a noisy city and live an efficient lifestyle. People's opportunities to get close to nature are gradually decreasing. At the same time, the health status of Chinese residents is also worrying; according to the big data of China's health released by China Digital Medical Network HC3i in 2014, China has more than 100 million people suffering from hypertension and hyperlipidemia [1], more than 70 million people are overweight, and the phenomenon of various diseases among young people shows an increasing trend.

Outdoor sport is an effective way to alleviate the above situation. Outdoor sports [2] can not only exercise our body but also help to cultivate our positive outlook on life and world outlook, stimulate our physical potential, strengthen our confidence to overcome difficulties, relieve psychological pressure, improve social communication ability, and enhance teamwork ability and cooperation spirit, which is very helpful to the improvement of people's comprehensive quality. Outdoor sport is a form of sports introduced into China from European and American countries in the 1980s. This kind of sports can not only meet the purpose of people's fitness and communication but also have a variety of ways for people to choose, such as adventure and relaxation outdoor sports. Outdoor sports can be carried out in a variety of natural environments, such as mountains, valleys, plateaus, deserts, and waters. There are many sports, and Americans often participate in more than 40. Facing so many outdoor sports, the primary problem faced by participants is how to choose the most suitable outdoor sports. The popularity of the Internet makes it easy for people to obtain a large amount of information. When outdoor sports lovers use the Internet to find the outdoor sports they want, due to the huge amount of information in the network, it reduces people's search efficiency, which is the problem of information overload [3]. Some Chinese tourism websites (such as Qunar, Ctrip, Tuniu, and Donkey mother) have some outdoor sports resources, but these websites focus on commercialization and cannot provide personalized recommendations for outdoor sports lovers. The information on Outdoor Sports Themed forums is not formatted, which is also not conducive to search. Search engines will not provide personalized search results. At present, the most effective way is to introduce recommendation system. The recommendation system can not only effectively alleviate the problem of information overload but also provide personalized recommendation services for users of the system, save users' time, improve users' search efficiency, and make people feel dependent on the recommendation system. At present, outdoor sports are becoming more and more popular in China, and the number of participants is also increasing. The sales of products related to outdoor sports are increasing rapidly, and the research literature related to outdoor sports is growing rapidly; on the other hand, the technology used in the recommendation system is becoming more and more mature. Moreover, from the search of CNKI (China National Knowledge Infrastructure) database, it can be seen that although there is research literature on tourism recommendation, so far there is no research literature on personalized recommendation for outdoor sports. With regard to recommendation algorithms, Najafabadi et al. [4] used a new graph-based structure to model the users' priorities and capture the association between users and items. Pereira et al. [5] studied cloud-based real-time collaborative filtering for item-item recommendations. Wei et al. [6] studied collaborative filtering and deep learning-based recommendation system for cold start items. Therefore, it is very necessary to carry out the research on personalized recommendation of outdoor sports and recommend personalized outdoor sports information for different users.

## 2. Pertinent Techniques

### 2.1. Recommendation System

The main purpose of the recommendation system is to recommend the user's preferred content to the user. If the recommendation system is abstracted and simplified, it can be divided into three modules (Figure 1): recommendation algorithm modeling, user modeling, and recommended item modeling. The simplification basis includes two aspects: for the establishment of user model, user information needs to be collected and processed, and for the recommendation target model, item object information needs to be collected and processed.

### 2.2. User Modeling

The quality of user modeling directly affects the accuracy, personalization, and recommendation efficiency of the recommendation system for users. Therefore, the user model should be able to dynamically and comprehensively express users' interests and preferences. Before modeling the users, the object to be modeled and content to be recommended should be clarified firstly. The modeling object in this paper is outdoor sport enthusiasts, and the recommendation content is outdoor sport item. Secondly, how to acquire the information and preference of users should be defined. Then, we conduct user modeling. The process of user modeling is shown in Figure 2. Collecting user information is very important for the recommendation system. In the recommendation system, there are two ways to obtain information: display and implicit. (1) We display the way to obtain information that can obtain the following types of data: ① the data provided by the user during registration, including the user's basic attributes, such as the user's name, income, occupation, age, native place, educational background, and family situation. The literature [7, 8] initializes the user modeling based on the user's basic attributes; ② data manually entered by the user, and the keywords entered by the user generally represent the user's preferred channel and theme; and ③ the user's explicit feedback data [9] show the user's evaluation of the viewed items, reflecting the user's liking for the items. Displaying the way to obtain user information can obtain user preferences more directly, truly, and accurately and can improve the quality of recommendation. The disadvantage of display acquisition method is that users need to spend time filling in information, which may cause users' resistance. The way of obtaining information depends on users, and the authenticity of the submitted information is closely related to the cooperation of users. (2) Implicit information acquisition methods include user implicit feedback data [10]. This method does not require users to actively submit their own information, but is obtained through users' behavior on the Internet. The implicit method of collecting user information cannot accurately determine the user's preferences. If the implicit tracking of users is excessive, it may reduce the user's experience. The advantage of implicit method is that the user does not need to display the submitted information, which saves the user's time of using the system, reduces the user's psychological burden, and improves the user's experience. The user information is used to represent the user; that is, the user is modeled. The representation method of the user model is as follows [11]:

#### 2.2.1. Vector Space Model

Vector space model uses feature vectors to represent users. Firstly, demographic attributes are used to extract keywords (or feature items) representing users. Each keyword represents a basic information of users and is given a weight. The user feature vector is generally represented by multiple keywords, and the formula is as follows:

(1) $$\begin{array}{c} \overset{⟶}{U_{u}}=\left\{K\left(k_{u}^{1},k_{u}^{2},k_{u}^{3},\ldots ,k_{u}^{n}\right),W\left(w_{u}^{1},w_{u}^{2},w_{u}^{3},\ldots ,w_{u}^{n}\right)\right\}, \end{array}$$

or

(2) $$\begin{array}{c} \overset{⟶}{U_{u}}=\left\{\left(k_{u}^{1},w_{u}^{1}\right),\left(k_{u}^{2},w_{u}^{2}\right),\left(k_{u}^{3},w_{u}^{3}\right),\cdots ,\left(k_{u}^{n},w_{u}^{n}\right)\right\}. \end{array}$$

Formulas (1) and (2) share the same principle, but differs from each other in form, where $\overset{⟶}{U_{u}}$ represents the characteristic vector of user *u*, *k*_*u*_^*n*^ represents the nth keyword of user *u*, and *w*_*u*_^*n*^ represents the weight of keyword *k*_*u*_^*n*^ of user *u* in user model.

#### 2.2.2. User-Item Ranking Model [12]

There is many corresponding information between users and projects. The display information includes users' scoring and purchase records, and the implicit information includes users' collection and browsing records. Scoring is used in this paper to model users and projects. In addition to the above two methods, there are other methods including topic representation method, keyword representation method, neural network representation method, topic representation method, case-based representation method, latent semantic index representation method, and content information representation method. The user modeling module also has the problems of user identification and user model update.

*(1) User identification*. User information collection is the first step of user modeling. Only after identifying [13] and confirming the user's identity can we obtain the information of a specific user. The methods of user identification include user cookie identification, login identification, and session identification.

*(2) User model update*. The user model of the recommendation system should be updated according to the feedback of system users and the evaluation of recommendation results [14], which will continuously improve the recommendation quality and accuracy of the recommendation system. The current updating technologies include adaptive neural network updating, updating according to the natural law of survival of the fittest, and adding new keywords to update.

### 2.3. Recommendation Content Modeling

In different application fields, the content objects recommended by the recommendation system are also different. From items on e-commerce websites to movies, news, and music, they all belong to the category of recommendation. However, different item objects have different attributes and characteristics, so the recommended objects cannot be modeled with unified standards. Combined with the description of recommendation target modeling in reference [15], when modeling the recommendation object, this paper refers to the user modeling method and the recommendation algorithm used, and then determines the recommendation target modeling method. If the feature vector method is used to model users and the content-based recommendation algorithm is combined, the corresponding feature vector should be used to model the recommended object; that is, the keyword of the recommended object with weight should be used (formula (3)). The recommendation object is divided into multiple categories, and the correlation degree between categories is calculated as the basis for recommendation.

(3) $$\begin{array}{c} \overset{⟶}{I_{i}}=\left\{K\left(k_{i}^{1},k_{i}^{2},k_{i}^{3}\ldots ,k_{i}^{n}\right),W\left(w_{i}^{1},w_{i}^{2},w_{i}^{3},\ldots w_{i}^{n}\right)\right\}. \end{array}$$

### 2.4. Recommendation Algorithm

In the recommendation system, the recommendation algorithm is the most core and key module. The quality of the recommendation algorithm directly affects the recommendation result and plays a decisive role in the performance of the recommendation system to a great extent. There are many kinds of recommendation algorithms, and the classification methods are slightly different. The recommendation algorithm used in this paper is shown in Figure 3.

#### 2.4.1. Collaborative Filtering Recommendation Algorithm

Collaborative filtering recommendation algorithm is the most widely used recommendation algorithm. There are many kinds of collaborative filtering recommendation algorithms, and the most widely used are user-based collaborative filtering recommendation algorithms [16] (UB-CF) and item-based collaborative filtering recommendation algorithms [17] (IB-CF). Both algorithms are based on user item scoring tables, and the difference can be understood as follows: UB-CF corresponds to “groups of people,” and IB-CF corresponds to “birds of a feather flock together.” The difference is that UB-CF seeks the similarity of rows and IB-CF seeks the similarity of columns.

*(1) User-based collaborative filtering*. The main idea of UB-CF is based on the assumption that users who score similar items also score similar items. In other words, if a user wants to get a recommendation, he needs to find a user similar to himself first.  Figure 4 shows the recommended schematic diagram of UB-CF, which describes the preferences of four users for four outdoor sports. It is found from user BCD that the preferences of user D are most similar to those of user A. In addition to the outdoor sports abc loved by user A, user D also likes outdoor sport d, so outdoor sport d is recommended to user A. As can be seen from the figure, UB-CF's recommendation is divided into three steps:

**Step 1 .**

Collect data.

The user item score matrix is generated according to the user's historical comment information. In addition to the user score, it can also include the user's browsing records, attention behavior, collection list, and click status. When collecting data, the data need to be denoised and normalized.

**Step 2 .**

Find close neighbors.

After obtaining the scoring matrix including target users, we calculate the similarity between target users and other users according to the similarity method and then take *K* similar users or take *δ* threshold nearest neighbor [19]. Similarity methods include the following: ① Jaccard coefficient; ② cosine similarity; ③ correlation similarity (Pearson's correlation coefficient); and ④ modified cosine similarity.

(1) Jaccard coefficient
  (4) $$\begin{array}{c} \text{sim}\left(u,v\right)=\frac{\left|N\left(u\right)\cap N\left(v\right)\right|}{\left|N\left(u\right)\cup N\left(v\right)\right|}, \end{array}$$
or
  (5) $$\begin{array}{c} \text{sim}\left(u,v\right)=\frac{\left|N\left(u\right)\cap N\left(v\right)\right|}{\sqrt{\left|N\left(u\right)\right|\left|N\left(v\right)\right|}}. \end{array}$$
Jaccard calculates the similarity of interest by using the items that have had positive feedback. *N* (*u*) represents the collection of items that have had positive feedback. Formula (4) is a simple calculation of Jaccard, and formula (5) is calculated by cosine similarity.
(2) Cosine similarity
  (6) $$\begin{array}{c} \text{sim}\left(u,v\right)=\cos\left(\overset{⟶}{u},\overset{⟶}{v}\right)=\frac{\overset{⟶}{u}\times \overset{⟶}{v}}{\left\|\overset{⟶}{u}\right\|\times \left\|\overset{⟶}{v}\right\|}, \end{array}$$
where $\overset{⟶}{u}\text{ and }\overset{⟶}{v}$ are the ranking vectors of user *u* and *v*, respectively.
(3) Correlation similarity
  (7) $$\begin{array}{c} \text{sim}\left(u,v\right)=\frac{\sum_{c\in I_{uv}}\left(R_{uc}-\bar{R_{u}}\right)\left(R_{vc}-\bar{R_{v}}\right)}{\sqrt{\sum_{c\in I_{uv}}{\left(R_{uc}-\bar{R_{u}}\right)}^{2}\sum_{c\in I_{uv}}{\left(R_{vc}-\bar{R_{v}}\right)}^{2}}}, \end{array}$$
where *I*_*uv*_ is the item that shares the same ranking of user *u* and *v*, $\bar{R_{u}}\text{ and }\bar{R_{v}}$ are the average rankings of user *u* and *v*, *c* is the ranking perspective of an item, and *R*_*uc*_ is the ranking of user *u* to item *c*.
(4) Modified cosine similarity
  (8) $$\begin{array}{c} \text{sim}\left(u,v\right)=\frac{\sum_{c\in I_{uv}}\left(R_{uc}-\bar{R_{u}}\right)\left(R_{vc}-\bar{R_{v}}\right)}{\sqrt{\sum_{c\in I_{u}}{\left(R_{uc}-\bar{R_{u}}\right)}^{2}\sum_{c\in I_{v}}{\left(R_{vc}-\bar{R_{v}}\right)}^{2}}}. \end{array}$$

The modified cosine similarity makes up for the defect that the cosine similarity is different in the user rating scale, and the symbol meaning is the same as the above formula.

**Step 3 .**

Generate recommendations.

In Step 2, the target user set or nearest neighbor set can be obtained, and the set is represented by *SN*_*u*_. Then, the user *u* scores that the item *i* on the *SN*_*u*_ is set as *P*_*ui*_. The calculation method of *P*_*ui*_ is as follows:

(9) $$\begin{array}{c} P_{ui}=\bar{R_{u}}+\frac{\sum_{n\in SN_{u}}\text{sim}\left(u,n\right)\cdot \left(R_{ni}-\bar{R_{n}}\right)}{\sum_{n\in SN_{u}}\left|\text{sim}\left(u,n\right)\right|}, \end{array}$$

where *sim* (*u*, *n*) represents the similarity between user *u* and *n*, and other symbols have the same meaning as the above formula. After calculating the evaluation diversity of items, we sort the evaluation diversity from high to low, generate top-N ranking [20], and recommend the best results to the target user.

*(2) Item-based collaborative filtering*. Item-based collaborative filtering (IB-CF) [21] was proposed by Sarwar et al. in 2001.  Figure 5 shows the schematic diagram of IB-CF recommendation principle. The diagram describes the preferences of four users for four outdoor sports. From the preferences of users, it can be seen that outdoor sports *a* is more similar to outdoor sport *c*, while user B likes outdoor sports *c*. Therefore, it is speculated that user B also likes outdoor sport *a* and recommends outdoor sport *a* to user B. General process of IB-CF first calculates the similarity between items to obtain the nearest neighbor set of the target user, calculate the similarity according to the user's score on the nearest neighbor set, and finally take the Top-N item to recommend to the target user according to the similarity. The method of calculating the similarity between items is basically the same as that of UB-CF.

UB-CF and IB-CF have their own advantages and disadvantages, which can be summarized as follows: UB-CF calculates the similarity between users through the scoring table of users and projects, and the recommended results are more accurate; the disadvantages are cold start and data sparsity; IB-CF generally adopts offline calculation, which is conducive to improving the real-time performance of the system. It is relatively advantageous in making recommendation explanation and the measurability of recommendation. The disadvantage is that the recommended items must have been commented, which is not conducive to discovering the potential interest of users. At the same time, there is also a cold start problem.

#### 2.4.2. Content-Based Filtering Recommendation Algorithms

As a long-standing algorithm, content-based recommendation [23] is applied in the field of feature engineering. The basic idea is to create relevant attribute portraits according to the content information of items. Taking Douban as an example, we first select the plot information of the movie as the portrait (assuming that users only watch specific types of movies); calculate the attribute similarity between the recommended object and the target movie; traverse the generated list; and select the movie with the largest similarity value of plot content. Finally, if the user does not watch the movie, we complete the recommendation; otherwise, we return to the previous operation. The specific implementation results of the recommendation strategy are shown in Figure 6. When the type of movie A is similar to that of movie C, the movie C with no connection is recommended to user a. In short, the core of the algorithm is to recommend items similar to their favorite items to users based on their own attributes.

As shown in Figure 7, taking outdoor sports as an example, user ABC has different preferences for outdoor sports abc. The spatial vector models of outdoor sports *a* and *c* have high similarity, while user A likes outdoor sport *a*, so outdoor sport c similar to outdoor sport *a* is recommended to user A.

There are four similarity calculation methods: Jaccard coefficient, cosine similarity formula, Dice coefficient, and TF-IDF formula. Among them, Jaccard coefficient and cosine similarity formula are the same as collaborative filtering. TF-IDF formula is as follows:

(10) $$\begin{array}{c} W\left(t,\bar{d}\right)=\frac{\left\{1+\;\log_{2}\left[tf\left(t,\bar{d}\right)\right]\right\}\times \;\log_{2}\left(N/n_{t}\right)}{\sqrt{{\sum_{t\in \bar{d}}\left[\left(1+\;\log_{2}\left(tf\left(t,\bar{d}\right)\right)\right)\times \;\log_{2}\left(N/n_{t}\right)\right]}^{2}}}, \end{array}$$

where $W\left(t,\bar{d}\right)$ is the weight of characteristic term *t* in document $\bar{d}$, $tf\left(t,\bar{d}\right)$ is the frequency of *t* occurs in document $\bar{d}$, and N is the total number of documents. Dice coefficient is similar with Jaccard, with the formula of:

(11) $$\begin{array}{c} \text{Dice}\left(A,B\right)=\frac{2\times \left|\text{keywords}\left(A\right)\cap \text{keywords}\left(B\right)\right|}{\left|\text{keywords}\left(A\right)\cup \text{keywords}\left(B\right)\right|}. \end{array}$$

This Dice coefficient only considers keywords and has no weight on keywords, so it is not suitable for weighted space vector model. Advantages of content-based recommendation [24]: users are relatively independent and high interpretability; the cold start of new items is better solved; the system responds quickly when calculating similarity offline. Disadvantages: feature extraction is relatively difficult, and it needs to be structured during storage. The novelty of recommendation is low, because the recommendation list is basically similar to the user's historical favorite items.

#### 2.4.3. Label-Based Recommendation Algorithm

Label [9, 20] is a keyword used to describe the nonhierarchical information of items [25]. Users' label items can not only enrich the description of items but also reflect users' interests and hobbies. One can use triples (*U*, *I*, *T*) similar to those above the data structure to represent user labeling (formula (0)).

(12) $$\begin{array}{c} \left(U,I,T\right)\left\{\left(U,I,T\right)|\left(U\left(u_{1},u_{2},\ldots u_{n}\right),I\left(i_{1},i_{2},\ldots ,i_{n}\right),T\left(t_{1},t_{2},\ldots ,t_{n}\right)\right)\right\}, \end{array}$$

where (*U*, *I*, *T*) indicates that the user *u* labels the article *i* with *t*, and uses the adjacency matrix to indicate that the user labels the article, 1 indicates that it is labeled, and 0 indicates that it is not labeled.

## 3. Critical Techniques

### 3.1. Cold Start

Historical data are an important basis for recommendation by the recommendation system. If the system lacks historical data, it will cause cold start [26]. In the personalized recommendation system for outdoor sports, the cold start problem refers to that there is no relevant information between users and outdoor sports after the development of the system. When the system administrator adds simulated user data and simulated outdoor sports project data to test the system, the system cannot effectively carry out personalized recommendation. The following ways are proposed in this paper to solve this problem, which is divided into three steps:

**Step 4 .**

When registering a new user in the system, in order to extract the effective information of the user, the system sets some user information as required items, such as user name, password, e-mail, education, income, age, marriage, gender, and the characteristics of liking outdoor sports. Through this part of information, the system can build the initial model of the new user.

**Step 5 .**

When the system administrator adds new outdoor sports, the characteristics, type, name, and introduction of outdoor sports are required. Through this information, the system can build the initial model of new outdoor sports.

**Step 6 .**

When the system has no associated information between users and outdoor sports, the system can use the user's initial model and the initial model of outdoor sports, use the similarity algorithm to calculate the similarity between users and outdoor sports, and then take the Top-N outdoor sports with the highest similarity to recommend to users.

After the system runs, there will be the related information of users and outdoor sports. At this time, when registering new users, in addition to using the above initial model to seek similar recommendations for users, collaborative filtering recommendation [24, 25] algorithm can also be added to seek similar recommendations [27], and the two similar recommendations can be combined for mixed recommendations.

On the premise that the system has the related information of users and outdoor sports, when adding new outdoor sports, the system can also recommend new outdoor sports to users by using the combination of initial model and collaborative filtering recommendation algorithm. When representing the feature vector of the user, the digital representation of the user feature is shown in Table 1.

### 3.2. Hybrid Recommendation Algorithm

Each recommendation algorithm has different principles, so its advantages and disadvantages, and recommendation results are also different. In order to make users get more efficient and accurate recommendations, we should absorb the advantages of multiple recommendation algorithms and avoid their own shortcomings. This is the most used hybrid recommendation algorithm at present. For example, adding content-based recommendation algorithm to collaborative filtering system can solve the sparsity problem of collaborative filtering. Of course, due to the characteristics of different application scenarios, the way of hybrid algorithm [28, 29] is also different. At present, there are several hybrid recommendation methods [27, 30], including weight combination, switch, mixed, feature combination, cascade combination, feature augmentation, and metal level.

Outdoor sport has its own uniqueness. In order to better recommend, the system will use the way of feature expansion and weighted combination to mix the collaborative filtering recommendation algorithm and content-based recommendation algorithm to form the final hybrid recommendation algorithm.

## 4. Collaborative Filtering Recommendation Algorithm Based on Extreme Residual Connection

In this chapter, the experimental details and experimental results of the content perception score prediction algorithm based on extreme residual connection proposed in this paper are introduced in detail. We explored on two real data sets ML-1m and ml-10m, and evaluated the experimental results by using the root-mean-square error evaluation index. Firstly, the experiments of three combination methods are carried out in the way of self-comparison to verify the ability of xRes connection to capture feature interaction and the necessity of constructing residual layer and transformation layer at the same time. Secondly, the effects of different parameters on the performance of the model are explored, and the network training and learning process is simulated. Finally, it makes a global comparison with other excellent seven methods and analyzes the recommendation performance of this study.

### 4.1. Performance Comparison of Network Component Combination Methods

A large-scale system is generally divided into multiple subsystems, and each subsystem corresponds to different functional modules of the system. At the beginning of system development, each subsystem will be divided to clarify the system architecture and design mode used. Before designing the personalized recommendation system for outdoor sports, the personalized recommendation model used by the system should be clear. To further compare the recommendation algorithms mentioned above, we explored the influence of xRes connection and pooling on the extraction of item feature vectors, and replaced them with the following two common methods selected in comparative experiments: xRConvCF-R (no conversion layer with residual layer) and xRConvCF-T (no residual layer with conversion layer). In order to avoid other components (such as word embedding layer and hidden layer) affecting the experimental analysis, we set all parameters in the model to the same value and only consider the new architecture formed by the combination of the two.

Figure 8 compares the training errors on two different data sets within 100 iterations of the three combined models. It can be found that the training error of xRConvCF is less than that of xRConvCF-T method on both data sets, which indicates the effectiveness of xRes connection to capture features. The root-mean-square error of xRConvCF is not significantly lower than that of xRConvCF-R, especially on ML-10m data set.

### 4.2. The Best Recommended Number *N* to Determine the Experiment

In order to determine the best recommendation number of the two recommendation algorithms, the best covering coefficient Φ is introduced above, selecting the recommended list lengths of 5, 10, 15, 20, 25, and 30 in turn, and making the Gini index curves of CF and CRGC-CF in the data sets MovieLens-100 k, MovieLens-latest-small, MovieLens-1 m, and MovieLens-10 m, respectively. As shown in Figure 9, the Gini index of the two algorithms both increases with the increase of the recommended list length *N*. The larger the data set, the smaller the scoring interval, and the stronger the diversity. As a whole, the recommendation algorithm optimized by covering rough granular computing model is better than the traditional collaborative filtering recommendation algorithm. The advantage is that insensitive to sparse data and has strong robustness. However, a certain amount of accuracy will be lost when the number of recommendations is too large. Hence, the most significance is that we should choose a moderate number of recommendations to get the best recommendation effect. The use case model of background management subsystem is shown in Figures 9 and 10. It can be found that energy efficiency increases with the increase of time under all the five recommendation algorithms, while energy efficiency reaches the maximum value under exhaustive searching and get the minimum value under GA algorithm.

### 4.3. Influence of Words Embedment Dimension on the Model

Figures 11 and 12 show the influence of the dimension of word embedding on the validation error of these methods on ml-1m and ml-10m data sets, respectively. Generally, with the increase of word vector embedding dimension, the verification error decreases first and then increases. The performance of the three models increases first and then decreases. As can be seen from the image, increasing the dimension from 50 to 100 can significantly improve the performance. When the dimension is too large, the performance decreases due to over fitting. However, with the increase of size, the increase of verification error is not obvious. Even when the dimension is 300, the performance is still within the acceptable range. This shows that the larger the embedded size of words, the stronger the representation ability. However, if the embedded size is too large, the complexity of our model will increase greatly. Therefore, we need to find the appropriate embedding size and strike a balance between performance and complexity.

## 5. Conclusions

This paper makes a beneficial attempt in the combination of outdoor sports and personalized recommendation technology, and the purpose of personalized recommendation of outdoor sports to users has been achieved. Therefore, the main work of this paper is as follows:

1. On the basis of user-based collaborative filtering recommendation algorithm (UB-CF), item-based collaborative filtering recommendation algorithm (IB-CF) and content-based recommendation algorithm (CBF), according to the characteristics of outdoor sports, this paper proposes to mix UB-CF, IB-CF, and CBF by means of feature expansion and weighted combination. The system adopts the hybrid recommendation model in actual recommendation. Aiming at the common cold start problem in the recommendation system, the system adopts CBF algorithm to solve the cold start problem of the system based on the characteristics of outdoor sports and the feature extraction of users and outdoor sports.
2. Based on the detailed demand analysis of the system, the system implementation is designed in detail, including system architecture, system function architecture, recommendation design, and database design. The development of personalized recommendation system for outdoor sports is completed, and the functions of hybrid recommendation model and system are realized.
3. The system adopts B/S architecture and front and rear end separated MVC three-tier design mode to develop a personalized recommendation system for outdoor sports, which effectively improves the performance of the system. Each functional module of the system is shown and described, and the hybrid recommendation model and corresponding code are described. The simulation data are used to test the system, and the results show that the system can effectively recommend users.

## Figures and Tables

**Figure 1:** Recommendation system model.

**Figure 2:** User modeling process.

**Figure 3:** Classification of recommendation algorithms.

**Figure 4:** Mechanism of UB-CF [18].

**Figure 5:** Mechanism of IB-CF [22].

**Figure 6:** Flowchart of content-based recommendation.

**Figure 7:** Item-based recommendation.

**Figure 8:** Error distribution.

**Figure 9:** Gini and the number of recommendations *N* of the two recommendation algorithms on different data sets.

**Figure 10:** Variation in number of layer II nodes according to queue I size.

**Figure 11:** Training error of the three models in ML-1m data set.

**Figure 12:** Training error of the three models in ML-10m data set.

**Table 1:** User characteristic number expression.

Age	Education experience	Income	Gender	Marriage	Number expression
Under 25	High school and below	2000 and below	Male	Married	1
26∼35	Junior college	2000∼4500	Female	Unmarried	2
36∼45	Undergraduate	4500∼7000			3
46∼55	Master	7000∼11000			4
Above 56	Doctor	Above 11000			5

## Data Availability

The data used to support the findings of this study are available from the corresponding author upon request.
